# Research on Subpixel Algorithm of Fixed-Point Tool Path Measurement

**DOI:** 10.1155/2021/7270908

**Published:** 2021-09-03

**Authors:** Xi Zhang, Zixie Guo, Xiangwei Liu, Longjia Zhang

**Affiliations:** School of Mechanical and Automation, Shanghai University, Shanghai 201900, China

## Abstract

Tool safety is an important part of machining and machine tool safety, and machine tool path image detection can effectively obtain the in-machine condition of a tool. To obtain an accurate image edge and improve image processing accuracy, a novel subpixel edge detection method is proposed in this study. The precontour is segmented by binarization, the second derivative in the neighborhood of the demand point is calculated, and the obtained value is sampled according to the specified rules for curve fitting. The point whose curve ordinate is 0 is the subpixel position. The experiment proves that an improved subpixel edge can be obtained. Results show that the proposed method can extract a satisfactory subpixel contour, which is more accurate and reliable than the edge results obtained by several current pixel-level operators, such as the Canny operator, and can be used in edge detection with high-accuracy requirements, such as the contour detection of online tools.

## 1. Introduction

With the continuous improvement of machining accuracy, especially precision machining, increasing tool chip parameters and optical imaging system precision is limited. Thus, under the same conditions, subpixel subdivision can improve measurement accuracy and reasonably control production cost. Therefore, examining a set of mature and stable subpixel contour detection algorithms is of considerable significance. This study conducts in-depth research on existing subpixel detection algorithms and proposes algorithm optimization for the environmental application of numerical control tools.

Image edge detection in computer image processing is a technology that was developed in the past but is continuously advancing. It plays a very important role in computer vision and image processing and is widely used in various fields such as image segmentation and pattern recognition [1, 2]. Feng et al. [3] proposed a saliency detection method based on the histogram contrast algorithm and wireless multimedia sensor network (WMSN) image to process animal images. In recent years, Zhang et al. [4] proposed an edge detection algorithm based on structured random forest, which can make full use of the RGB-D image information of Kinect. With the development of industrial cameras and the improvement of image quality, the application of image edge detection technology in the industry became increasingly extensive.

Early commonly used pixel-level edge extraction methods are mainly classical edge extraction operator algorithms, such as the Sobel operator [5], Scharr operator [6], Laplacian operator [7–10], and gate operator. These algorithms demonstrate one-pixel accuracy; that is, they can determine which pixel the edge is in and the most accurate position, which traditional algorithms cannot judge. With the improvement of the accuracy requirements of target edge detection, the pixel-level edge obtained by common operators cannot meet the needs of precision measurement and visual calibration. Therefore, research on subpixel edge detection is essential. Current subpixel detection methods include the probability theory method, demodulation measurement method, and polynomial interpolation method [11–16].

Subpixel algorithms have been studied by many people. Wu proposed a subpixel edge detection algorithm based on Franklin's matrix, which was fast and accurate and demonstrated strong noise immunity [17]. Xie et al. [18] proposed an improved subpixel edge detection algorithm combining coarse positioning with fine positioning. Kumar and Ratnam [19] used the moment invariant subpixel detection method to improve the detection accuracy. A tool wear measurement system based on machine vision was developed to solve the problems of manual operation and shutdown detection in actual production [20]. Wu proposed a laser image subpixel edge detection method based on Gabor filtering and mathematical morphology [21]. Ai et al. proposed a corner detection algorithm based on subpixel edges [22].

## 2. Materials and Methods

Image subpixel processing involves complex mathematical operations, which can considerably increase the running time of a program and affect the efficiency of the entire production and processing. In actual NC machining, the fixed-point tool diameter is typically used as a parameter. Fixed-point tool diameter measurement is employed to determine the diameter of a tool by measuring the radial distance at the fixed height of the tool.

In this situation, subpixel processing the entire image is not necessary, we only need to process the image to obtain the pixel-level contour of the image, then establish the ROI region within the specified line range, and use a specific subpixel algorithm for the ROI region to obtain the required subpixel points, which can take into account the improvement of calculation accuracy and algorithm efficiency at the same time.

### 2.1. Image Preprocessing

Image preprocessing is an important part of finding the image edge point, but images before being processed may be affected by uncertainty and/or inaccuracy, so sometimes we need a fuzzy preprocessing [23, 24]. Image preprocessing and ROI region positioning in advance can realize the fast positioning of the subpixel region. In this study, the reverse binarization operation is performed on the image to distinguish the image foreground and background before determining the ROI region. The calculation method is shown in equation (1). The advantage of this method is that because the contour envelope algorithm used in contour extraction will envelope the white region, the reverse binarization of the image can reduce the influence of image boundary on image contour extraction.

(1) $$\begin{array}{c} dst\left(x,y\right)=\left\{\begin{array}{c} 0,\\ \text{Maxval,} \end{array}\;\right.\begin{array}{c} \;i\text{f }src\left(x,y\right)>\text{threshold},\\ \text{otherwise.} \end{array} \end{array}$$

As the input image is a binary image and its value is only 0 and 255, in the image processing, the input image is binary *f*(*i*, *j*) when scanning, and scanning is terminated in the following two cases: (1) *f*(*i*, *j* − 1) = 0 and *f*(*i*, *j*) = 255, where *f*(*i*, *j*) is the starting point of the outer boundary, and (2) *f*(*i*, *j*) = 255 and *f*(*i*, *j* + 1) = 0, where *f*(*i*, *j*) is the starting point of the hole boundary. This contour extraction algorithm comes from a paper published by Satoshi Suzuki [25].

At this time, the starting point is determined, and the contour boundary sequence can be obtained with the Freeman chain code [26]. However, the actual image may generate multiple contours owing to the influence of a backlight, but the cutter part occupies the dominant position in the image contour. Therefore, the longest contour sequence is screened so as to successfully separate the tool contour from the contour extracted from the picture.

After the image contour sequence is obtained, the next step involves finding the fixed point in the contour sequence to measure the position of the pixel-level contour points in the contour sequence. In this study, to find the one-dimensional sequence, a binary search algorithm is used to search for the contour points. First, the known array is sorted by the quick sort algorithm. Second, the binary search method is used for the search.

As the data structure of points belongs to user-defined data structures, the sorting rules must be defined in the quick sort algorithm. In this study, the ascending order of the *Y* coordinate and the ascending order of the *X* coordinate are chosen when the *y* coordinate is the same to sort the contour points. This method places the contour points on the same row of pixels arranged from left to right, which can provide a satisfactory basis for searching.

According to the search method described above, when the first contour point in the line where the measurement position is located is detected, all points with the same *y* coordinate as the point are taken out, and the two points with the smallest and largest *X* coordinate are taken as the two starting positions of the fixed-point tool path subpixel iteration; the region formed by extending 10 pixels to the left and right with these two points as the center is the ROI region where the subpixel points in the target row are located as shown in Figures 1and 2 .

If the gray value at the back of the falling-edge or rising-edge ROI is insufficient, then the ROI will be extended 5 pixels backward until the value is insufficient. If the gray value at the front of the rising-edge or falling-edge ROI is insufficient, then the ROI will be extended 5 pixels forward until the value is insufficient.

### 2.2. Single-Point Subpixel Algorithm

In the common image edge solving methods, finding the highest point of the first derivative and finding the zero-crossing point of the second derivative are the two common methods. As shown in Figure 3, the black coordinate points represent the derivative values obtained by solving the first derivative of the image with Canny operator. The blue curve is the result of interpolating these values. It can be seen that the maximum value of the interpolation curve is between the black coordinate points, which means that the actual maximum value is not on the coordinate points, and the actual edge of the image is also on the subpixel points. In this study, the second derivative is used to calculate the single-point subpixel.

Assume that the image function expression of the ROI region is *f*(*x*), and the expression of the first derivative is

(2) $$\begin{array}{c} f^{\prime }\left(x\right)=\;\underset{h⟶0}{\lim}\frac{f\left(x\;+\;h\right)-\;f\left(x\right)}{h}. \end{array}$$

The image function expression is discretized, and the pixel interval *h* = 1 is taken, and then the discretized second-derivative expression is as follows:

(3) $$\begin{array}{c} f^{\prime \prime }\left(x\right)=\;f^{\prime }\left(x\;+\;1\right)-\;f^{\prime }\left(x\right). \end{array}$$

After expansion, the second-order expression is as follows:

(4) $$\begin{array}{c} f^{\prime \prime }\left(x\right)=f\left(x+2\right)-2f\left(x+1\right)+f\left(x\right). \end{array}$$

Thus, the convolution kernel of the second-order differential operator can be obtained as follows:

(5) $$\begin{array}{c} \left[1,-2,1\right]. \end{array}$$

After the image function of the one-dimensional ROI is convoluted with the convolution kernel of the second-order differential operator, the second-order difference value can be obtained, as shown in Figure 4.

It can be found from Figure 4 that the curve distribution near the highest point and the lowest point of the curve composed of second-order derivative values is similar to the quartic function curve. At the same time, it is noted that the zero-crossing point is not at the pixel point, but at the subpixel point, which indicates that the image edge is also at the subpixel point. In this study, we approximately replace the second-derivative curve of the gray value with the quartic curve.

Suppose that the expression of the quartic curve is

(6) $$\begin{array}{c} f\left(x\right)=ax^{4}+bx^{3}+cx^{2}+dx+e, \end{array}$$

where *a*, *b*, *c*, *d*, and *e* are constant and *a*≠0.

By solving the root of the above quartic equation, the zero-crossing point of the second derivative of gray value in the ROI region can be obtained.

The quartic curve zero-crossing problem can be transformed into the solution of the root of the quartic equation of one variable. Finding the root of a high-order equation is tedious; thus, the numerical solution can be obtained by the iterative method. In this study, the Durand–Kerner (D–K) algorithm [27] is selected to solve the problem. For the quaternary equation with one variable, the complex numbers *P*, *Q*, *R*, and *S* are assumed to be the roots of equation (7). After decomposition, the following equation can be obtained:

(7) $$\begin{array}{c} f\left(x\right)=\left(x-P\right)\left(x-Q\right)\left(x-R\right)\left(x-S\right). \end{array}$$

For all of the *X*'s, we can factor out the values from this.

(8) $$\begin{array}{c} P=x-\frac{f\left(x\right)}{\left(x-Q\right)\left(x-R\right)\left(x-S\right)}. \end{array}$$

The corresponding fixed-point iteration formula is as follows:

(9) $$\begin{array}{c} x=x_{0}+\frac{f\left(x_{0}\right)}{\left(x_{0}-Q\right)\left(x_{0}-R\right)\left(x_{0}-S\right)}, \end{array}$$

where *x*_0_ ≠ *Q*, *R*, and *S*.

If the approximate points of *Q*, *R*, and *S* are substituted, that is, *q* ≈ *Q*, *p* ≈ *P*, and *s* ≈ *S*, then *P* remains a fixed point. Therefore, the general form of the iterative formula for finding the root can be expressed as follows:

(10) $$\begin{array}{c} x_{k+1}=x_{k}+\frac{f\left(x_{k}\right)}{\left(x_{k}-q\right)\left(x_{k}-r\right)\left(x_{k}-s\right)}. \end{array}$$

Through iteration, the values of *P*, *Q*, *R*, and *S* can be obtained. In practical application, we only need the values that meet the requirements, so the values of *P*, *Q*, *R*, and *S* need to be filtered according to the definition of zero-crossing point:

1. The zero-crossing point must be a real root, and its imaginary part is 0
2. The value of the root of the zero crossing should be within the axis interval of *x* where the maximum and minimum values are located

If the obtained values do not meet the above conditions, it is deemed that the calculation of subpixel edge points at this point has failed; if there is a root that meets the above conditions, take it as the coordinate of the subpixel edge point in the ROI area coordinate system and map it to the image coordinate system through the following equation:

(11) $$\begin{array}{c} x_{n}=x_{o}-l+x_{s}+x_{r}-1, \end{array}$$

where *x*_*n*_ is the value of the subpixel point under the global coordinate of the image, *x*_*o*_ is the value of the initial test pixel point under the global coordinate of the image, *x*_*s*_ is the value of the first fitting-point pair in the ROI, *x*_*r*_ is the value of the subpixel point under the ROI coordinate system, and *l* is the extended length of the pixel's value forward.

Through equation (6), we can find that at least five different points must be fitted to determine the constant value in the expression. In order to make the change trend of the fitting curve closer to the reality, first select the two points where the maximum and minimum values of the second-order difference value are located in the second-order difference ROI area and then expand from these two points; the two points near each of these two points are selected to form a group of six-point fitting-point pairs. However, in the actual calculation, only one point may exist between the maximum and minimum values. Therefore, the constant value solution methods can be divided into five- and six-point methods.

For five-point methods, assume that the position of the fitting point in the ROI is defined as the axis data of *x*-axis, and its corresponding second-order difference value is the axis data of the *y*-axis. It can be converted into the following matrix expression after being placed in the point pair:

(12) $$\begin{array}{c} \left[\begin{array}{ccccc} x_{1}^{4} & x_{1}^{3} & x_{1}^{2} & x_{1} & 1\\ x_{2}^{4} & x_{2}^{3} & x_{2}^{2} & x_{2} & 1\\ x_{3}^{4} & x_{3}^{3} & x_{3}^{2} & x_{3} & 1\\ x_{4}^{4} & x_{4}^{3} & x_{4}^{2} & x_{4} & 1\\ x_{5}^{4} & x_{5}^{3} & x_{5}^{2} & x_{5} & 1 \end{array}\right]\left[\begin{array}{c} a\\ b\\ c\\ d\\ e \end{array}\right]=\left[\begin{array}{c} y_{1}\\ y_{2}\\ y_{3}\\ y_{4}\\ y_{5} \end{array}\right]. \end{array}$$

For convenience, the above equation can be simplified as *AX* = *B*. As the *A* matrix is a full-rank matrix, the matrix is invertible; thus, the expression can be solved by the following formula:

(13) $$\begin{array}{c} X=A^{-1}B, \end{array}$$

where *X* is the constant value to be solved.

Similarly, the matrix of the six-point fitting method can be expressed by a matrix similar to the matrix of the five-point fitting method in the equation (12). For convenience, the matrix solution equation of the six-point fitting method can be expressed as *AX* = *B*. As the *A* matrix is not a square matrix, it cannot be solved simply in the form of an inverse matrix, but the numerical solution of the Eu matrix can be obtained with the least squares estimation method. Therefore, the value of Eu can be obtained as

(14) $$\begin{array}{c} X={\left(A^{T}A\right)}^{-1}A^{T}B. \end{array}$$

At this point, the expression of the quartic curve can be obtained using the five- or six-point fitting method.

### 2.3. Algorithm Framework

The whole subpixel algorithm is shown as Algorithm1.

Finally, the *X* coordinates of subpixel edge points in the original image *x*_*n*_ can be obtained by the above algorithm, combined with the fixed measurement position height, that is, the fixed *Y* coordinates *y*_*m*_, and we can get subpixel point (*x*_*n*_, *y*_*m*_).

## 3. Results and Discussion

To verify the correctness and accuracy of the algorithm, experimental analysis is conducted by using actual tool photos and comparing the Canny operator, binary algorithm, and subpixel algorithm [28] proposed by Rafael Grompone von Gioi.

### 3.1. Experimental Environment

The algorithm is tested in a laboratory environment and in Shanghai, Xuzhou, Suzhou, and other processing plants. The test results show that a Haas machine tool and tools for an actual shooting machine environment are used in the test.

A photo of the tools is presented in Figure 5.

The preprocessed image is presented in Figure 6.

### 3.2. Verification

#### 3.2.1. Five-Point Method

Suppose that the 112th-row pixel of the tool image is measured at a fixed point, and one of the binary contour edge coordinates is obtained after binarization. The ROI area is obtained by extending 10 pixels forward and backward from this point, and the gray value of the ROI is as follows:

(15) $$\begin{array}{c} \left[248,247,246,245,243,239,225,192,138,82,44,23,14,9,7,7,7,6,6,6\right]. \end{array}$$

Thus, it can be determined that the gray change type is a falling-edge, and the value of its corresponding position after the second-order difference is as follows:

(16) $$\begin{array}{c} \left[0,0,0,-1,-2,-10,-19,-21,-2,18,17,12,4,3,2,0,-1,1,0,0\right]. \end{array}$$

The maximum value of the second-order difference is 18 at the 10th position, the minimum value is −21 at the 8th position, and the number of intermediate points is 1. Therefore, a point is taken from both sides of the maximum value to form a five-point sequence [−19, −21, −2, 18, 17]. Next, the fitting coordinate system is established according to the position and second-order difference value, and the five-point sequence is transformed into Table 1.

According to the sequence of fitting points, the coefficient matrix of the quartic curve can be obtained by solving the equations with the least squares method.

(17) $$\begin{array}{c} {\left[-0.0833,-2.5,27.583,-66,22\right]}^{T}. \end{array}$$

Therefore, the quartic curve expression is as follows:

(18) $$\begin{array}{c} f\left(x\right)=-0.00833x^{4}-2.5x^{3}+27.583x^{2}-66x+22. \end{array}$$

The position relationship between the fitting-point and quartic curve expression is shown in Figure 7.

By solving the matrix equation and according to the coordinate transformation formula, the subpixel coordinates of a single point can be updated to (227.087, 112).

#### 3.2.2. Six-Point Method

In the early stage of the procedure, similar to the five-point method, the pixel is selected as [91, 110].

The ROI is obtained by extending 10 pixels forward and backward from this point. The gray value of the ROI is as follows:

(19) $$\begin{array}{c} \left[254,253,247,238,231,226,219,199,160,107,59,30,17,12,10,9,9,8,8,7\right]. \end{array}$$

And the value of its corresponding position after the second-order difference is as follows:

(20) $$\begin{array}{c} \left[0,-5,-3,2,2,-2,-\mathrm{13},-\mathrm{19},-\mathrm{14},5,\mathrm{19},\mathrm{16},8,3,1,1,-1,1,-1,1\right]. \end{array}$$

In the fitting coordinate system, the six-point sequence is transformed into Table 2.

According to the sequence of fitting points, the coefficient matrix of the quartic curve can be obtained by solving the equations with the least squares method.

(21) $$\begin{array}{c} {\left[3.167,-17.505,-0.785,2.551,-0.3125\right]}^{T}. \end{array}$$

The quartic curve expression is as follows:

(22) $$\begin{array}{c} f\left(x\right)=3.167x^{4}-17.505x^{3}-0.785x^{2}+2.551x-0.3125. \end{array}$$

The D-K algorithm [26] is used to solve the root of the quartic equation. The numerical results of the iterative process are as shown in Table 3.

After 16 iterations, the numerical solution is obtained. According to the screening conditions of the zero-crossing point, the fourth root of the quartic equation solution is selected as the position of the zero-crossing point. According to the coordinate transformation formula, the coordinates of a single-point subpixel can be updated to (89.793, 110), and its position is shown in Figure 8. On the right side is the binary edge point, and on the left side is the subpixel edge point calculated by the algorithm.

### 3.3. Comparison

In order to verify the accuracy of this algorithm, we also carried out many comparative experiments and selected some common image edge algorithms to compare with the algorithms in this paper. In the experiment, different algorithms are used to find the image edge points in the specified area of the same tool picture. Some experimental results are as follows.

A total of 16 pairs of points are selected for comparison, and the area is shown as Figure 9.

The image *Y*-axis is 195–210 pixels, and the left figure's *X*-axis is 220–233 pixels, and the right figure's *X*-axis is 779–791 pixels, respectively.

Binarization, the Canny operator, the subpixel algorithm proposed by Rafael Grompone von Gioi [28], and the algorithm in this study are used to process the region. The data obtained are shown in Table 4.

Through the values of edge points obtained by different algorithms in Table 4, combined with the pixel coordinates in Figure 9, we can draw the following conclusions:

1. Binarization and Canny operator can only feedback pixel-level image edge point coordinates. Both this algorithm and R-algorithm can provide subpixel level edge point coordinates.
2. Combined with the pixel coordinates in Figure 9, we can find that the image edge effect obtained by binarization is the worst, and both the algorithm in this paper and R-algorithm can provide better image subpixel edge points.

## 4. Conclusions

The experimental data can prove that this algorithm can indeed improve the pixel-level edge points to subpixel level edge points. The subpixel points obtained by the proposed method demonstrate high accuracy and are tested in a tool machining environment, which can help increase the accuracy of tool diameter measurement.

## Figures and Tables

**Figure 1:** Grayscale map of the ROI region of fixed-point measurement (falling-edge).

**Figure 2:** Grayscale map of the ROI region of fixed-point measurement (rising-edge).

**Figure 3:** First-order derivative curve of gray value in the ROI region.

**Figure 4:** Second-derivative curve of gray value in the ROI region.

**Figure 5:** Flat bottom knife picture.

**Figure 6:** Preprocessed image.

**Figure 7:** Fitting curve.

**Figure 8:** Subpixel edge points.

**Figure 9:** The test figure.

**Algorithm 1:** Subpixel algorithm.

**Table 1:** Coordinates of fitting points.

Point	*P*1	*P*2	*P*3	*P*4	*P*5
Coordinate	**(1,** −**19)**	**(2,** −**21)**	**(3,** −**2)**	**(4, 18)**	**(5, 17)**

**Table 2:** Coordinates of fitting points.

Point	*P*1	*P*2	*P*3	*P*4	*P*5	*P*6
Coordinate	**(1, −13)**	**(2, −19)**	**(3, −14)**	**(4, 5)**	**(5, 19)**	**(6, 16)**

**Table 3:** Iterative process of root.

Number of iterations	*P*	*Q*	*R*	*S*
1	−19.372 − 2.547*i*	1.512 + 5.553*i*	−8.754 + 6.415*i*	−3.407 − 4.349*i*
2	73.797 − 61.853*i*	1.290 + 6.074*i*	−1.691 − 7.623*i*	−2.230 − 4.324*i*
3	35.058 − 8.776*i*	−0.755 + 11.781*i*	−11.648 + 1.478*i*	−2.4134 − 5.867*i*
…	—	—	—	—
15	26.58 − 6.136*e*^−91^*i*	6.537 − 1.473*e*^−90^*i*	0.525 + 0*i*	3.461 − 2.286*i*
**16**	**26.588** **+** **0*i***	**6.537** **+** **0*i***	**0.525** **+** **0*i***	**3.461** **+** **0*i***

**Table 4:** Comparative data.

Binarization	Canny	R-subpixel	Text subpixel
[229, 195]	[226, 195]	[226.243, 195]	**[226.272, 195]**
[229, 196]	[227, 196]	[225.884, 196]	**[225.803, 196]**
[227, 197]	[226, 197]	[225.334, 197]	**[225.145, 197]**
[226, 198]	[225, 198]	[224.87, 198]	**[224.778, 198]**
[226, 199]	[225, 199]	[224.521, 199]	**[224.514, 199]**
[226, 200]	[224, 200]	[224.313, 200]	**[224.316, 200]**
[226, 201]	[224, 201]	[224.228, 201]	**[224.237, 201]**
[226, 202]	[224, 202]	[224.243, 202]	**[224.214, 202]**
[226, 203]	[224, 203]	[224.418, 203]	**[224.398, 203]**
[226, 204]	[225, 204]	[224.746, 204]	**[224.694, 204]**
[227, 2051	[225, 205]	[225.231, 2051	**[225.046, 2051**
[229, 206]	[226, 206]	[225.949, 206]	**[225.889, 206]**
[229, 207]	[227, 207]	[226.686, 207]	**[226.445, 207]**
[229, 208]	[227, 208]	[227.187, 208]	**[227.239, 208]**
[229, 209]	[227, 209]	[227.33, 209]	**[227.306, 209]**
[229, 210]	[227, 210]	[227.362, 210]	**[227.328, 210]**
[783, 195]	[785, 195]	[784.971, 195]	**[784.414, 195]**
[783, 196]	[785, 196]	[785, 196]	**[784.475, 196]**
[783, 197]	[785, 187]	[785, 197]	**[784.515, 197]**
[783, 198]	[785, 198]	[785, 198]	**[784.454, 198]**
[783, 199]	[785, 199]	[784.986, 199]	**[784.487, 199]**
[783, 200]	[785, 200]	[784.986, 200]	**[784.453, 200]**
[783, 201]	[785, 201]	[784.985, 201]	**[784.515, 201]**
[783, 202]	[785, 202]	[784.971, 202]	**[784.389, 202]**
[783, 203]	[785, 203]	[784.971, 203]	**[785.042, 203]**
[783, 204]	[785, 204]	[785, 204]	**[784.47, 204]**
[783, 205]	[785, 205]	[784.986, 205]	**[784.505, 205]**
[783, 206]	[785, 206]	[784.971, 206]	**[784.51, 206]**
[783, 207]	[785, 207]	[784.985, 207]	**[784.504, 207]**
[783, 208]	[785, 208]	[785, 208]	**[784.504, 208]**
[783, 209]	[785, 209]	[785, 209]	**[784.504, 209]**
[783, 210]	[785, 210]	[784.987, 210]	**[784.454, 210]**

## Data Availability

The data used to support the findings of this study are available from the corresponding author upon request.
